The article "Twist1 accelerates tumour vasculogenic mimicry by inhibiting Claudin15 expression in triple‐negative breast cancer" was retracted in 2024. Reasons: plagiarized images; duplicated images; overlap with other authors' work; unreliable data.

# Twist1 accelerates tumour vasculogenic mimicry by inhibiting Claudin15 expression in triple‐negative breast cancer

**DOI:** 10.1111/jcmm.15167

**Published:** 2020-05-29

**Authors:** Danfang Zhang, Baocun Sun, Xiulan Zhao, Huizhi Sun, Jindan An, Xian Lin, Dongwang Zhu, Xueming Zhao, Xudong Wang, Fang Liu, Yanhui Zhang, Jiameng Liu, Qiang Gu, Xueyi Dong, Zhiqiang Qiu, Zhiyong Liu, Hong Qi, Na Che, Jing Li, Runfen Cheng, Xu Zheng

**Affiliations:** ^1^ Department of Pathology Tianjin Medical University Tianjin China; ^2^ Department of Pathology General Hospital of Tianjin Medical University Tianjin China; ^3^ Department of Pathology Cancer Hospital of Tianjin Medical University Tianjin China

**Keywords:** angiogenesis, claudin15, triple‐negative breast cancer, Twist1, vasculogenic mimicry

## Abstract

The up‐regulation of EMT regulator Twist1 has been implicated in vasculogenic mimicry (VM) formation in human triple‐negative breast cancer (TNBC). Twist1 targets the Claudin15 promoter in hepatocellular carcinoma cells. Claudin family members are related with TNBC. However, the relationship between Claudin15 and VM formation is not clear. In this study, we first found that Claudin15 expression was frequently down‐regulated in human TNBC, and Claudin15 down‐regulation was significantly associated with VM and Twist1 nuclear expression. Claudin15 down‐regulation correlated with shorter survival compared with high levels. Claudin15 silence significantly enhanced cell motility, invasiveness and VM formation in the non‐TNBC MCF‐7 cells. Conversely, an up‐regulation of Claudin15 remarkably reduced TNBC MDA‐MB‐231 cell migration, invasion and VM formation. We also showed that down‐regulation of Claudin15 was Twist1‐dependent, and Twist1 repressed Claudin15 promoter activity. Furthermore, GeneChip analyses of mammary glands of Claudin15‐deficient mice indicated that Claudin18 and Jun might be downstream factors of Twist1‐Claudin15. Our results suggest that Twist1 induced VM through Claudin15 suppression in TNBC, and Twist1 inhibition of Claudin15 might involve Claudin18 and Jun expression.

## 1 INTRODUCTION

Breast cancer is the most frequent malignancy among women worldwide.^1^ Triple‐negative breast cancer (TNBC) cells do not express oestrogen receptor (ER), progesterone receptor (PR) or human epidermal growth factor receptor 2 (HER2)^2^ and account for 15‐26% of breast cancer cases.^3^, ^4^ TNBC cases show significant differences in incidence, survival and response to therapy compared with non‐TNBC cases. The prognosis of patients with TNBC is worse compared with that of patients with other breast cancer subtypes because of the unique genotype and clinical behaviour of TNBC.^2^ TNBCs are more aggressive than other breast cancer subtypes and have a higher tendency to metastasize to visceral organs. Endocrine therapy, anti‐HER2 antibody and chemotherapy have no effect on TNBCs.^5^ Despite ongoing clinical trials, an efficacious treatment for patients with TNBC is not yet available.^6^, ^7^, ^8^, ^9^ The molecular mechanisms of TNBC development need to be investigated to help establish a better treatment strategy.^6^

The article "Twist1 accelerates tumour vasculogenic mimicry by inhibiting Claudin15 expression in triple‐negative breast cancer" was retracted in 2024. Reasons: plagiarized images; duplicated images; overlap with other authors' work; unreliable data.

Six molecular subtypes of breast cancer have been identified:^10^, ^11^ Claudin‐low, luminal A, luminal B, HER2‐enriched, basal‐like and a normal breast‐like group.^11^, ^12^ Claudin‐low breast cancer is the most recently identified subtype.^10^ This distinct subtype is characterized by the low gene expression of tight junction proteins Claudins 3, 4 and 7, and E‐cadherin and the high gene expression of epithelial‐to‐mesenchymal transition (EMT)‐associated molecules.^10^ The Claudin family is comprised of 27 members that function as integral membrane proteins,^13^ ranging in size from 22 to 27 kDa.^14^ Claudins belongs to the four transmembrane protein class containing the carboxyl‐terminus in the cytoplasm and two extracellular loops.^15^ Claudins links to occludins and junctional adhesion molecules to form the backbones of tight junctions.^14^ Claudins have also been found to be altered in several cancers.^16^, ^17^, ^18^ However, the full Claudin expression profile and functions in different tumours are still not well characterized.^16^

Tumour progression is angiogenesis‐dependent. Anti‐angiogenic agents are important strategy in malignant cancer treatment.^19^, ^20^ Vasculogenic mimicry (VM) reflects the vascularization of malignant tumours, a process involving the generation of microvascular channels by tumour cells.^21^ VM channels are formed by tumour cells but not by endothelial cells. VM occurs in many aggressive tumours such as melanoma, inflammatory breast carcinoma, prostate carcinoma, ovarian carcinoma, hepatocellular carcinoma and gastrointestinal stromal tumours.^22^, ^23^, ^24^, ^25^, ^26^, ^27^ Tumours with VM are more aggressive, and patients with VM have a poorer prognosis than those without VM.^28^, ^29^, ^30^ Increasing evidence indicates that EMT is essential in VM formation.^26^ EMT‐inducing transcription factors, including Slug, Twist1, Zinc finger E‐box binding homeobox 2 (ZEB2) and bone morphogenetic protein 2 (BMP2), are associated with VM existence in different malignant tumours.^26^, ^31^, ^32^, ^33^ We previously demonstrated that hypoxia induces VM through accelerating Twist1 expression in TNBC.^32^ Moreover, we found that Twist1 bound to the Claudin15 promoter in hepatocellular carcinoma cells.^34^ Based on these results, in this study we examined the hypothesis that Twist1 binds to Claudin15 promoter to inhibit its expression to promote VM formation.

The article "Twist1 accelerates tumour vasculogenic mimicry by inhibiting Claudin15 expression in triple‐negative breast cancer" was retracted in 2024. Reasons: plagiarized images; duplicated images; overlap with other authors' work; unreliable data.

## 2 MATERIAL AND METHODS

### 2.1 Reagents and cell culture

The human breast cancer cell lines MCF‐7 and MDA‐MB‐231 were cultured in RPMI‐1640 medium with 10% FBS, 4 mM L‐glutamine and 1% penicillin‐streptomycin. Matrigel (BD Bioscience) was diluted with RPMI‐1640 medium. The primary antibodies used in this study are listed in Table S1. All secondary antibodies were purchased from Zhongshan Golden Bridge Biotechnology Co., Ltd.

### 2.2 Patient samples

The Tianjin General Hospital Ethics Committee approved the human studies. All clinical investigations were conducted according to the principles stated in the Declaration of Helsinki. The patients were informed of the aims, methods and other details of the present study. We collected samples from 90 patients with breast cancer with detailed pathological and clinical information. All patients underwent surgery in Tianjin General Hospital from 1997 to 2004. The median age of the patients was 51.0 years (31 to 74 years). All patients had invasive breast cancer, and axillary node metastases were present in 24 patients. The diameter of the primary tumour in four patients was < 2 cm and > 5 cm in 15 patients. The follow‐up period started at the time of the surgery and ended in December 2008.

### 2.3 Immunohistochemical staining

Formalin‐fixed, paraffin‐embedded tissues were sectioned, dewaxed and rehydrated using graded concentrations of alcohol. Endogenous peroxidase was blocked using 5% goat serum at room temperature for 10 minutes. The sections were heated in a microwave oven in citrate buffer for 20 minutes. The slides were incubated with primary antibodies overnight at 4°C, washed with PBS, and individually incubated with biotin‐labelled or FITC‐labelled secondary antibodies. The colour was developed using DAB. The sections were counterstained with haematoxylin or DAPI and observed using a microscope (80i, Nikon). Staining was scored using the previously published method.^32^ Briefly, positive tumour cells were categorized as follows: 0 = undetectable, 1 = weak, 2 = moderate and 3 = strong. The number of positive cells out of 100 tumour cells per field was visually evaluated and scored as follows: 0 < 10% positive, 1 < 25%, 2 < 50% and 3 > 50%. The staining index or the sum of the staining intensity and the positive cell score were used to determine the result for each sample. A sample was defined as positive when the staining index was > 1. VM and endothelial vessels were counted at 400 × magnification, and the score for each sample was defined as the average of 10 fields of view.

The article "Twist1 accelerates tumour vasculogenic mimicry by inhibiting Claudin15 expression in triple‐negative breast cancer" was retracted in 2024. Reasons: plagiarized images; duplicated images; overlap with other authors' work; unreliable data.

### 2.4 Periodic acid Schiff (PAS) double staining

After immunohistochemical analysis of sections for CD31 expression, the sections were exposed to 1% sodium periodate for 10 minutes, washed for 5 minutes in distilled water and then incubated for 15 minutes with PAS at 37°C. The sections were counterstained with haematoxylin and observed using a microscope (80i, Nikon).

### 2.5 Expression plasmids and RNA interference

The full‐length Twist1 complementary cDNA was amplified using PCR from a library of normal human embryo cDNA digested with XhoI/EcoRI and subcloned into pcDNA3.1 vectors.^26^ The constructs were confirmed by DNA sequencing. A small interfering RNA (siRNA) kit (pGP‐Twist1‐shRNA) was purchased from GenePharm. The target sequence was 5´‐AAGCTGAGCAAGATTCAGACC‐3´ (siTwist1 nucleotides 505‐525).^26^ An expression clone datasheet of Claudin15 (EX‐V1637‐Lv201) was purchased from GeneCopoeia. A Claudin15 siRNA kit (HSH006369‐1‐LVRU6MP) was purchased from GeneCopoeia. The target sequence was 5′‐CTGTGGAAACCTTTGGCTT‐3′. A non‐silencing siRNA sequence (targeting 5′‐AATTCTCCGAACGTGTCACGT‐3′) was used as a negative control.

### 2.6 Luciferase reporter gene assays

The GLuc‐ON Claudin15 Promoter Reporter Clone Datasheet was purchased from GeneCopoeia. Transactivation assays were performed with the Dual‐Luciferase Reporter Assay System (Promega). Cotransfection of MCF‐7 cells was performed by percutaneous ethanol injection, and cells were cultured in a 3D Matrigel system for 72 h. Luciferase activities were measured with the Synergy 2 microplate reader system (Gene).

### 2.7 Western blotting

Lysates were prepared using a buffer containing 1% SDS, 10 Mm Tris‐HCl, pH 7.6, 20 μg/mL aprotinin, 20 μg/mL leupeptin and 1 mM AEBSF. The protein concentration of lysates was measured using the Bradford method. Approximately 20 µg of protein was separated on an 8% SDS‐PAGE gel and electroblotted onto a PVDF membrane. After blocking with 5% fat‐free milk in TBS‐Tween overnight, the membrane was incubated with primary antibodies overnight at 4°C. After washing with TBS‐Tween three times, the membrane was labelled with horseradish peroxidase‐conjugated anti‐goat IgG (1:1000) for 1 hours at room temperature. Blots were developed using a DAB kit, GAPDH was used as an internal control, and the bands were analysed using a gel imaging system (Kodak).

### 2.8 Generation of Claudin15‐deficient mice

The targeting vector was constructed using two overlapping clones encoding mouse Claudin15 with 5 exons picked up from a 129/Sv genomic library (Figure 5A and 5B).^35^ Two potential targeted clones (2C7, 5E11) were identified by Southern blotting. Both were expanded and frozen. Southern blotting analysis was conducted by a 5′ probe and Neo‐probe. The strategy is shown in Figure 5A. The genomic DNA of the potential clones 2C7 and 5E11 was digested by Nde I and analysed by Southern blot for 5′ probe using forward primer 5′‐TGATGCTCCACTCTGTGAACCCTG‐3′ and reverse primer 5′‐CTGAATGCCTTGCATCTTCCTGAG‐3′. The genomic DNA of the potential clones 2C7 and 5E11 was digested by BamHI and analysed by Southern blot for Neo‐probe using forward primer 5′‐CCTGAATGAACTGCAGGACGAGG‐3′ and reverse primer 5′‐AGCTCTTCAGCAATATCACGGGTAGC‐3′.

The article "Twist1 accelerates tumour vasculogenic mimicry by inhibiting Claudin15 expression in triple‐negative breast cancer" was retracted in 2024. Reasons: plagiarized images; duplicated images; overlap with other authors' work; unreliable data.

### 2.9 RT‐PCR

Total RNA of mammary glands in Claudin15‐deficient mice was isolated using TRIzol reagent (Invitrogen Life Technologies) and reverse transcribed (TaKaRa Biotechnology Co., Ltd). Conventional and quantitative reverse‐transcription polymerase chain reactions (RT‐PCRs) were performed using primers as follows: mouse Claudin15 forward primer 5′‐CATCTTTGAGAACCTGTGGTACAGC‐3′ and reverse primer 5′‐GATGGCGGTGATCATGAGAGC‐3′. GAPDH was the control, and the primers were as follows: forward primer 5′‐CCTGGCCAAGGTCATCCATGAC‐3′ and reverse primer 5′‐TGTCATACCAGGAAATGAGCTTG‐3′.

### 2.10 GeneChip and data analysis

Total RNA of mice mammary gland was isolated by the TRIZOL, and the RNA integrity was assessed using Agilent Bioanalyzer 2100 (Agilent Technologies). The sample labelling, microarray hybridization and washing were performed based on the manufacturer's standard protocols. Briefly, total RNA was transcribed to double strand cDNA, and then synthesized cRNA and labelled with biotin. The labelled cRNAs were hybridized onto the microarray. After washing and staining, the arrays were scanned by the Affymetrix Scanner 3000 (Affymetrix). Affymetrix GeneChip Command Console (version 4.0, Affymetrix) was used to analyse array images to get raw data. Next, GeneSpring software (version 12.5; Agilent Technologies) was used to finish the basic analysis with the raw data. Differentially expressed genes were then identified through fold change as well as *P* value calculated with t test. The threshold set for up‐ and down‐regulated genes was a fold change ≥ 2.0 and a *P* value ≤ .05. Afterwards, GO analysis and KEGG analysis were applied to determine the roles of these differentially expressed mRNAs. Finally, hierarchical clustering was performed to display the distinguishable genes’ expression pattern among samples. Real‐time PCR was performed to validate the selected differentially expressed genes using LightCycler^®^ 480 II (Roche). The primers are listed in Table S2. Furthermore, protein interactions in the Claudin15‐deficient mammary glands were obtained using the online database resource ‘Search Tool for the Retrieval of Interacting Genes’ (STRING 10.0). Only interactions with the highest confidence score (0.800 and above) were used to build networks using Cytoscape.

The article "Twist1 accelerates tumour vasculogenic mimicry by inhibiting Claudin15 expression in triple‐negative breast cancer" was retracted in 2024. Reasons: plagiarized images; duplicated images; overlap with other authors' work; unreliable data.

### 2.11 Statistical analysis

SPSS version 11.0 was used to evaluate the data. The chi‐square test was performed to assess the pathological and clinical characteristics of the TNBC and non‐TNBC groups. The survival of these two groups was evaluated using Kaplan‐Meier analysis. The chi‐square test was also performed to assess the expression of different proteins expression of the VM‐positive and VM‐negative groups. The relationships between VM, Twist1, VE‐Cadherin and Claudin15 were analysed by correlation analysis. The two‐tailed Student's *t* test was performed to compare the parameters between two groups. Statistical significance was defined as *P* < .05.

## 3 RESULTS

### 3.1 Pathological and clinical features of TNBC

We collected samples from 90 breast cancer patients and categorized samples as TNBC based on expression of ER, PR and HER2 using immunohistochemistry (IHC). The TNBC tumours had small, poorly differentiated and highly mitotic tumour cells, and necrosis was present in the centre of the tumour nests. Table S1 summarizes the pathological and clinical features of the patients in each group. The median ages at diagnosis of patients in the TNBC and non‐TNBC groups were 47 and 51 years, respectively. The median survival of all patients was 80.0 months. The survival rate of the non‐TNBC group was 87.3%, whereas that of the TNBC group was 61.8%. The mean survival times of the non‐TNBC and TNBC groups were 135.1 ± 4.94 months and 88.4 ± 7.43 months, respectively (*χ* ^2^ = 15.683, *P* = .001).

IHC staining of CD31 indicated that the microvessel density of the TNBC patients was higher compared with that of the non‐TNBC patients (Figure S1B,C, respectively; *t* = 2.956, *P* = .038). VM channels that did not express CD31 but stained with PAS (Figure S1B) were identified in approximately 37.5% of the TNBC group and in 16.0% of the non‐TNBC group (Figure S1B, Table S3; *χ* ^2^ = 5.225, *P* = .022). There was a significant difference in the expression of Claudin15 and nuclear Twist1 between the TNBC and non‐TNBC groups. Low expression of Claudin15 and high expression of nuclear Twist1 were detected in the TNBC group (Table S2).

Kaplan‐Meier survival analysis shows that the survival of VM‐positive patients was worse than that of VM‐negative patients (Figure 1A; *χ* ^2^ = 1.460, *P* = .227), and the survival of Claudin15‐negative patients was worse than that of Claudin15‐positive patients (Figure 1B; *χ* ^2^ = 4.766, *P* = .029).

The article "Twist1 accelerates tumour vasculogenic mimicry by inhibiting Claudin15 expression in triple‐negative breast cancer" was retracted in 2024. Reasons: plagiarized images; duplicated images; overlap with other authors' work; unreliable data.

**Figure 1:** Kaplan‐Meier survival analysis of human breast cancer. A, Overall survival of VM + and VM‐ breast cancer. B, Overall survival of Claudin15 + and Claudin15‐ breast cancer. C, Overall survival of Twist1 + and Twist1‐ breast cancer. D, Overall survival of VE‐cadherin + and VE‐cadherin‐ breast cancer

### 3.2 The relationship between Claudin15, Twist1 and VE‐cadherin expression and VM in human breast cancer

Approximately 66.7% of VM‐positive TNBC patients expressed low levels of Claudin15, and 24% of VM‐negative TNBC patients expressed high levels of Claudin15 (*χ* ^2^ = 9.789, *P* = .002; Table 1 and Figure 2). Approximately 86.7% of VM‐positive TNBC patients expressed high levels of Twist1 in the plasma, and 36.4% of VM‐negative TNBC patients expressed low levels of Twist1 in the plasma (*χ* ^2^ = 7.071, *P* = .008; Table 1 and Figure 2). Approximately 73.3% of VM‐positive TNBC patients expressed high levels of VE‐cadherin, and 20.0% of VM‐negative TNBC patients expressed low levels of VE‐cadherin (*χ* ^2^ = 5.838, *P* = .016; Table 1 and Figure 2). Pearson correlation analysis indicated that Claudin15 expression was negatively correlated with VM and plasma and nuclear Twist1 expression, and the relationships are significant (Table 2).

**Table 1:** The differences of Claudin15, cytoplasmic Twist1, nuclear Twist1 and VE‐Cadherin expression between VM‐positive and VM‐negative groups in TNBC

Factors	VM (−)	VM (+)	*χ* ^2^	*P*
Claudin15				
（−）	6	10	9.789	.002**
（+）	19	5		
Cytoplasmic Twist1				
（−）	16	2	7.071	.008**
（+）	9	13		
Nuclear Twist1				
（−）	22	8	3.095	.079
（+）	3	7		
VE‐Cadherin				
（−）	20	4	5.838	.016*
（+）	5	11		

* *P* ≦ .05; **P ≦ .01; ***P ≦ .001

**Figure 2:** Claudin15, Twist1 cytoplasm, Twist1 nuclear and VE‐Cad expression in VM‐positive and VM‐negative groups in TNBC patients. The expressions of Claudin15, Twist1 cytoplasm, Twist1 nuclear and VE‐Cad in VM‐positive and VM‐negative groups of TNBC patients. The ruler is 100 μm

**Table 2:** The correlation of VM, Twist1, VE‐Cadherin and Claudin15 in breast cancer

Factors	*r*	*P*
VM	−.339	.001***
Cytoplasmic Twist1	−.236	.089
Nuclear Twist1	−.291	.027*
VE‐Cadherin	−.175	.224

* Means *P* < .05, **Means *P* < .01, ***Means *P* < .001.

### 3.3 Twist1 leads to VM formation through inhibition of Claudin15 transcription

To investigate the relationship between Twist1, Claudin15 and VM in breast cancer, we modulated the levels of Twist1 expression by overexpression (in non‐TNBC MCF‐7 cells) or shRNA‐based techniques (in TNBC MDA‐MB‐231 cells). The results of 3D cell culture indicated that MDA‐MB‐231‐shTwist1 cells failed to form VM channels on Matrigel, and there were more VM channels in the MCF‐7‐Twist1 cells compared with the control group (Figure 3A). MCF‐7‐Twist1 cells also showed a significantly increased migration ability (Figure 3B,C). We observed an up‐regulation of Claudin15 expression in the MDA‐MB‐231‐shTwist1 cells compared with the control group and decreased Claudin15 expression in the MCF‐7‐Twist cells (Figure 3D,F). In the process of VM formation by tumour cells, VE‐cadherin plays an important role as an intercellular adhesion and cascade signal transduction molecule.^26^, ^36^ There was also a significant change in VE‐cadherin in these two groups (Figure 3D,F).

The article "Twist1 accelerates tumour vasculogenic mimicry by inhibiting Claudin15 expression in triple‐negative breast cancer" was retracted in 2024. Reasons: plagiarized images; duplicated images; overlap with other authors' work; unreliable data.

**Figure 3:** Twist1 leading to VM formation through inhibition of Claudin15 transcription. A, The effect of Twist1 expression on VM channel formation. VM channels in 3D cell culture of MDA‐MB‐231‐shTwist1 cells and MCF‐7‐Twist1 cells. B, Wound healing assays of MDA‐MB‐231‐shTwist1 cells and MCF‐7‐Twist1 cells. C, Quantification of wound healing of MCF‐7‐Twist1 cells and MDA‐MB‐231‐shTwist1 cells (n = 3). D, Western blotting of Claudin15 expression and VE‐cadherin in the indicated cells. E, Dual‐luciferase reporter assays in MCF‐7 cells cotransfected with a Claudin15 luciferase reporter and Twist1 expression vector. F, The expression and quantifications of Twsit1, Claudin15 and VE‐cadherin in the different groups. Arrows indicated the positive signals. The ruler is 100 μm, and the error bar indicates the standard error of mean (SEM). *P < .05, **P < .01, ***P < .001

We previously found that Twist1 could bind and inhibit the promoter of Claudin15. To examine whether a similar mechanism was present in breast cancer cells, we performed luciferase assays using MCF‐7 cells cotransfected with a Claudin15 promoter‐luciferase construct and Twist1 expression vector. Twist1 overexpression resulted in an approximate fivefold transactivation inhibition of Claudin15 promoter activity (Figure 3E). These results suggest that the Claudin15 promoter is also a target of Twist1 binding in breast cancer cells.

### 3.4 Claudin15 up‐regulation leads to decreased MDA‐MB‐231 breast cancer cell invasion, migration and VM formation in vitro

Given the inhibitory effect of Twist1 on Claudin15, we next examined the effect of Claudin15 up‐regulation on VM formation, wound healing and cell invasion of TNBC. The expression of Claudin15 was lower in TNBC MDA‐MB‐231 cells compared to higher levels in non‐TNBC MCF‐7 cells. We used an in vitro model of 3D culture for investigating tube formation to evaluate whether Claudin15 mediates VM formation of TNBC cells. The results indicated that both MDA‐MB‐231‐Claudin15 and MCF‐7 cells failed to form typical circle‐like structures on the 3D Matrigel medium (Figure 4A). Wound healing assay and the quantitative analysis demonstrated that the up‐regulation of Claudin15 inhibited the migration of MDA‐MB‐231 cells, while Claudin15 down‐regulation accelerated the speed of wound healing of MCF‐7 cells (Figure 4B‐D). Moreover, in the Matrigel invasion assay presented in Figure 4E,F, a decrease in cell invasion was observed in the Claudin15‐transfected MDA‐MB‐231 cell line compared with the negative vector control, and there was increased invasion in MCF‐7‐shClaudin15 cells compared with the control.

The article "Twist1 accelerates tumour vasculogenic mimicry by inhibiting Claudin15 expression in triple‐negative breast cancer" was retracted in 2024. Reasons: plagiarized images; duplicated images; overlap with other authors' work; unreliable data.

**Figure 4:** Claudin15 up‐regulation leads to decreased MDA‐MB‐231 breast cancer cell invasion, migration and VM formation in vitro. A, 3D culture in both MDA‐MB‐231 and MCF‐7 cells up‐regulated or down‐regulated for Claudin15 expression on the 3D Matrigel medium (n = 3). B, Wound healing assays of MDA‐MB‐231 and MCF‐7 cells. C, Quantitative analysis of wound healing of MCF‐7 and MCF‐7‐shClaudin15 cells (n = 3). D, Quantitative analysis of wound healing of MDA‐MB‐231 and MDA‐MB‐231‐Claudin15 cells (n = 3). E, Matrigel invasion assays of MDA‐MB‐231‐Claudin15 and MCF‐7‐shClaudin15 cells compared with the control. F, Quantitative analysis of invasion assays (n = 3). E, The Matrigel invasion assay. F, Western blotting of VE‐cadherin, E‐cadherin and Vimentin. The ruler is 100 μm, and the error bar indicates the standard error of mean (SEM). *P < .05, **P < .01, ***P < .001

VE‐cadherin, E‐cadherin and Vimentin are the most frequently reported markers of TNBC and VM formation. MDA‐MB‐231‐Claudin15 cells expressed lower VE‐cadherin than the MDA‐MB‐231 controls, while down‐regulation of Claudin15 in MDF‐7 cells increased the expression of it. MDA‐MB‐231‐Claudin15 cells expressed higher E‐cadherin and Vimentin than the MDA‐MB‐231 controls, while down‐regulation of Claudin15 in MDF‐7 cells inhibited the expression of them (Figure 4G).

### 3.5 Morphology of mammary glands in Claudin15‐deficient mice

To explore the biological function and downstream molecules of Claudin15 in breast tumours, we constructed a targeting vector to disrupt the Claudin15 gene by replacing exon 1 with the neomycin‐resistance gene (Figure 5A,B). Heterozygous mice were crossed into C57BL/6 wild‐type mice through more than 5 generations and interbred to produce homozygous mice. Claudin15 was not detected in the small intestine of homozygous mutant mice by immunoblotting as well as RT‐PCR (Figure 5C,D). H&E staining indicated that there was hyperplasia in the mammary glands of Claudin15^−/−^ mice (Figure 5E).

**Figure 5:** Generation of Claudin15^−/−^ mice. A, Construction of the wild‐type allele, the targeting vector and the targeted allele of the Claudin15^−/−^ mice. B, Final targeting vector. C, Southern blot analysis of the targeted clones. 5′ probe: The genomic DNA of the potential clones 2C7 and 5E11 was digested by Nde I and analysed by Southern blot for a 14 kb band from wild‐type allele and a 9.1 kb band from recombinant allele; 2C7 and 5E11 were positive. Neo‐probe: The genomic DNA of the potential clones 2C7 and 5E11 were digested by BamHI and analysed by Southern blot for a 9.8 kb band from the recombinant allele; 2C7 and 5E11 were positive. D, Loss of Claudin15 mRNA in the mammary gland of Claudin15‐deficient mice by RT‐PCR. GADPH is the control. E, H&E staining of Claudin15^−/−^ mice and wild‐type mice. Compared with the mammary gland of wild‐type mice, there was hyperplasia in the mammary glands of Claudin15^−/−^ mice

The article "Twist1 accelerates tumour vasculogenic mimicry by inhibiting Claudin15 expression in triple‐negative breast cancer" was retracted in 2024. Reasons: plagiarized images; duplicated images; overlap with other authors' work; unreliable data.

### 3.6 Deletion of Claudin15 gene caused phenotype change of mammary glands

To investigate the phenotype change of mammary glands, we performed GeneChip assays and the differentially expressed genes were identified. Gene set enrichment analysis (GSE‐A) was performed on all differentially expressed genes to determine the top canonical pathways associated with Claudin15 deletion. The top enriched genes (*P* < .05), identified from the training set used to predict the validation set, are displayed in a heat map in Figure 6A. Table S4 lists the 73 differentially expressed genes between Claudin15^−/−^ mammary glands and Claudin15^+/+^ mammary glands. KEGG analysis showed that expressions of these genes involved in cell junction signalling pathways have significantly changed, such as focal adhesion, gap junction, regulation of actin cytoskeleton, ECM‐receptor interaction and tight junction (Figure 6B). Real‐time PCR results indicated that mRNA expressions of Claudin18, trp53inp1, Jun and Ddit4 were significantly up‐regulated in the Claudin15^−/−^ mammary glands (Figure 6C). The STRING online database predicted the protein interaction in the Claudin15‐deficient mammary glands. The results revealed a predicted interaction between Claudin18, Jun and Claudin15 (Figure S2).

**Figure 6:** Identification and validation of differentially expressed genes between Claudin15^−/−^ and Claudin15^+/+^ type mammary glands. A, Differentially expressed genes between Claudin15^−/−^ and Claudin15^+/+^ type mammary glands. The top enriched genes (*P* < .05), identified from the training set used to predict the validation set, are listed in a heat map. B, Enrichment analysis of pathways for differentially expressed genes. Pathway analysis was predominantly based on the KEGG database. *P* values < .05 using the chi‐square test were indicated as statistically significant. C, Verification of differentially expressed genes between Claudin15^−/−^ and Claudin15^+/+^ type mammary glands. The error bar indicates the standard error of mean (SEM). *P < .05

The article "Twist1 accelerates tumour vasculogenic mimicry by inhibiting Claudin15 expression in triple‐negative breast cancer" was retracted in 2024. Reasons: plagiarized images; duplicated images; overlap with other authors' work; unreliable data.

## 4 DISCUSSION

We examined the clinical and pathological features of Claudin15‐expressing human breast cancers, and the results indicated that Claudin15 expression was negatively correlated with VM, VM‐related proteins and EMT‐inducing transcription mediator Twist1 in TNBC. Furthermore, we addressed the repression of Twist1 on Claudin15 transcription and the promotion of VM by the down‐regulation of Claudin15 in vitro*.* To investigate the downstream molecule of Claudin15, GeneChip was used to identify the differentiated expressed genes between mammary glands in the Claudin15‐deficient mice and those in the wide type mice.

Breast cancer represents multiple disease types due to different molecular fingerprints.^12^ Claudin‐low breast tumours are mostly TNBC, and these cancers are characterized by down‐regulation of Claudin family members.^10^, ^12^, ^37^ Claudins 1, 3, 4, 5 and 7 have proven involvement in human breast cancers.^17^, ^18^ IHC confirmed that expressions of Claudin1 and 7 were absent or markedly decreased in the majority of invasive breast carcinomas as compared with normal ducts of mammary gland.^18^ Conversely, the protein expression levels of Claudins 3, 4 and 5 were significantly increased in breast neoplasia.^17^, ^38^ Low level of Claudin1 and high levels of Claudin 3 and 4 were associated with poor prognosis in TNBC.^17^, ^39^ In the present study, we found that Claudin15 was detected at low levels in TNBC. Kaplan‐Meier survival analysis showed that the survival of Claudin15‐negative patients was worse than that of Claudin15‐positive patients. Hence, low expression of Claudin15 might be an independent marker of poor prognosis in breast cancers.

The function of Claudins in different tumour development is highly tissue‐specific and regulated by the exact tumour microenvironment.^16^ The loss of Claudins and the related tight junctions leads to the loss of cell adhesion and cell polarity,^40^ and serves as an important step in EMT and tumour metastasis. Down‐regulation of Claduin1 in breast cancer facilitated the tumour development, and Claudin4 protein expression was decreased in primary and metastatic pancreatic cancer,^41^ which reduces invasiveness of these cells.^42^ Conversely, some Claudins, such as Claudin2, 3 and 4 in breast cancer, are expressed at a high level and promote tumour metastasis. Claudin2 engages with integrin to facilitate mouse breast tumour cells adherence to extracellular matrix (ECM) components and proliferation in the metastatic sites.^43^ Overexpression of Claudin3 and 4 in TNBC is a compensation for disruption of Claudin1, which results in an increase in invasion, motility, and cell survival.^44^ Here, VM is another independent marker of poor prognosis in breast cancers. The negative relation between Claudin15 level and VM existence suggested that loss of Claudin15 and promotion of VM formation is the cause of poor prognosis in breast cancer.

The article "Twist1 accelerates tumour vasculogenic mimicry by inhibiting Claudin15 expression in triple‐negative breast cancer" was retracted in 2024. Reasons: plagiarized images; duplicated images; overlap with other authors' work; unreliable data.

Since VM has been identified in more than 10 malignant tumours, it has been widely associated with large tumour size, aggressive type, higher TNM stage and higher metastasis or recurrence frequency in different tumours.^29^ There are several potential mechanisms for the anti‐angiogenic treatment resistance.^45^, ^46^, ^47^ Tumours with VM are not sensitive to anti‐angiogenic agents targeting endothelial cells.^32^ Tumour cells lining VM channels express some endothelial cell markers including factor VIII, Laminin5 and VE‐cadherin.^21^, ^48^ Epithelial tumour cells acquire the ability to form VM. This process involves a transition from the epithelial feature to endothelial phenotype, which is similar to that of EMT. Transcription factors Twist1, Slug, ZEB1 and ZEB2 induce expression of EMT markers, such as VE‐cadherin, Vimentin and ß‐catenin, in hepatocellular carcinoma and colon cancer.^26^, ^31^, ^33^, ^49^ Claudin‐low breast cancers show the morphological features of EMT, and the molecular characterization of Claudin‐low tumours includes the enrichment of EMT‐inducing factors such as Snail, Slug, Twist1, Twist2, ZEB1 and ZEB2.^37^ The Claudin promoters contain binding sites for EMT‐inducing mediators. Snail and Slug bind to the E‐box motifs of Claudin1 to disrupt tight junctions in human breast cancer cell lines.^50^ We identified a negative correlation between Claudin15 and the EMT‐inducing Twist1 and EMT marker VE‐cadherin. We previously demonstrated that Twist1 could bind to the Claudin15 promoter. These results suggested that Twist1 might control the transcription of Claudin15 in TNBC.

According to data from human breast cancer, we regulated Twist1 and Claudin15 expression in TNBC cell MDA‐MB‐231 and non‐TNBC cell MCF‐7. Twist1 overexpression in MCF‐7 cells enhanced tumour cell mobility and VM formation, and also inhibited Claudin15 expression. Knock‐down of Twist1 in MDA‐MB‐231 cells resulted in increased Claudin15 expression and loss of VM channel formation on Matrigel. Our luciferase assays demonstrated that Twist1 inhibited promoter activity of Claudin15. Moreover, silencing of Claudin15 in MCF‐7 cells promoted VM formation and VE‐cadherin expression. These data suggest that Twist1 accelerated VM formation through inhibiting Claudin15 transcription in TNBC. The involvement of Twist1 in VM formation was first reported in hepatocellular carcinoma. Hypoxia induced Twist1 and bcl‐2 to form a complex and synergistically activate the transcriptional activity of VE‐cadherin, which led to VM and tumour promotion.^34^ These data suggest that Twist1 induces VM formation through different signalling pathways in specific niches.

The article "Twist1 accelerates tumour vasculogenic mimicry by inhibiting Claudin15 expression in triple‐negative breast cancer" was retracted in 2024. Reasons: plagiarized images; duplicated images; overlap with other authors' work; unreliable data.

Claudin15 is a member of the Claudin family that is expressed in lung, heart, gut, muscle and thymus of mice.^35^ Claudin15 is required for fusion of multiple lumen into a single gut lumen in zebrafish.^51^ Deficiency of Claudin15 in mice gut epithelium can cause morphogenesis by disordered fluid accumulation.^35^ In this study, we show for the first time an involvement of Claudin15 in breast cancer development and VM formation. Claudin15‐deficient mice showed hyperplasia in the mammary glands. GeneChip analyses identified 73 differentially expressed genes between Claudin15^−/−^ mammary glands and Claudin15^+/+^ mammary glands. These genes are involved in several pathways important for tumour angiogenesis and metastasis, including focal adhesion signalling pathway, gap junction signalling pathway, regulation of actin cytoskeleton signalling pathway, ECM‐receptor interaction signalling pathway and tight junction signalling pathway. Furthermore, STRING online database predicted the putative protein‐protein interactions between Claudin18 and Jun with VM‐associated factor E‐cadherin and EMT translational factor Yes‐associated protein 1 (YAP1).^52^ The results suggested that Claudin18 and Jun might be the downstream effectors of Twist1‐mediated inhibition of Claudin15 transcription.

In conclusion, we showed for the first time that Claudin15 was correlated with TNBC VM formation and that the Twist1 and Claudin15 pathway potentially regulates VM formation. Twist1 induced VM through the suppression of Claudin1 transcriptional activity, and Twist1‐inhibited Claudin15 promoter activation might involve Claudin18 and Jun expression. Our findings provide a molecular basis for the role of EMT mechanism in TNBC VM formation. Twist1, Claudin15 and related molecular pathways might be used as novel therapeutic targets for the inhibition of TNBC angiogenesis and metastasis.

## CONFLICT OF INTEREST

The authors declare no conflict of interest.

## AUTHOR CONTRIBUTIONS

Baocun Sun was responsible for conception, design and final approval of the version to be published. Danfang Zhang and Xiulan Zhao involved in conception, design, animal experiment and drafted the manuscript. Xiulan Zhao and Dongwang Zhu were responsible for IHC staining, PAS/CD31 double staining and taking pictures. Xueming Zhao, Xudong Wang, Zhiqiang Qiu and Jindan collected the data of breast cancer patients and analysed the data. Fang Liu, Na Che and Xueyi Dong made the sections and tissue blocks for mice model. Huizhi Sun, Jing Li and Xian Lin involved in the animal treatment and data collection of animal experiment. Jiameng Liu and Hong Qi carried out Western blot and participated in animal experiment. Xu Zheng and Yanhui Zhang were responsible for cell culture in vitro. Runfen Cheng and Zhiyong Liu participated in IF staining. All authors read and approved the final manuscript.

The article "Twist1 accelerates tumour vasculogenic mimicry by inhibiting Claudin15 expression in triple‐negative breast cancer" was retracted in 2024. Reasons: plagiarized images; duplicated images; overlap with other authors' work; unreliable data.

## Supporting information

Fig S1

Fig S2

Table S1

Table S2

Table S3

Table S4
